# Novel Radiomics Features for Automated Detection of Cardiac Abnormality in Patients with Pacemaker

**DOI:** 10.1155/2022/1279749

**Published:** 2022-05-05

**Authors:** M. Umesh Pai, Ali Abbasian Ardakani, Aditya Kamath, U. Raghavendra, Anjan Gudigar, Naveen Venkatesh, Jyothi Samanth, Tom Devasia, Mukund A. Prabhu, Niranjana Sampathila, G. Muralidhar Bairy

**Affiliations:** ^1^Department of Cardiovascular Technology, Manipal College of Health Professions, Manipal Academy of Higher Education, Manipal 576104, India; ^2^Department of Radiology Technology, School of Allied Medical Sciences, Shahid Beheshti University of Medical Sciences, Tehran, Iran; ^3^Department of Biomedical Engineering, Manipal Institute of Technology, Manipal Academy of Higher Education, Manipal 576104, India; ^4^Brown University, Providence, Rhode Island 02912, USA; ^5^Department of Instrumentation and Control Engineering, Manipal Institute of Technology, Manipal Academy of Higher Education, Manipal 576104, India; ^6^Department of Cardiology, Kasturba Medical College, Manipal Academy of Higher Education, Manipal 576104, India

## Abstract

Cardiac pacemakers are used in the treatment of patients with symptomatic bradycardia. The pacemaker paces the heart at the predetermined rate to maintain uninterrupted cardiac activity. Usually, pacemaker lead will be connected to the right atrium (RA) and right ventricle (RV) in dual-chamber pacemaker implantation and RV alone in single-chamber pacemaker implantation. This alters the route of proper conduction across the myocardial cells. The cell-to-cell conduction transmission in pacing delays the activation of selected intraventricular myocardial activation. Pacing-induced cardiomyopathy (PICM) is most commonly defined as a drop in left ventricle ejection fraction (LVEF) in the setting of chronic, high-burden right ventricle (RV) pacing. Currently, very few effective treatments are standard for PICM which rely on the detection of the RV pacing. Such treatments have primarily focused on upgrading to cardiac resynchronization therapy (CRT) when LVEF has dropped. However, the early and accurate detection of these stress factors is challenging. Cardiac desynchrony and interventricular desynchrony can be determined by various echocardiographic techniques, including M-mode, Doppler method, tissue Doppler method, and speckle tracking echocardiography which is subjective measures and shows a significant difference between RV and LV preejection period where the activation of LV is delayed considerably. Computer-aided diagnosis (CAD) is a noninvasive technique that can classify the ultrasound images of the heart in pacemaker-implanted patients and healthy patients with normal left ventricular systolic function and further detect the variations in pacemaker functions in its early stage using heart ultrasound images. Developing such a system requires a vast and diverse database to reach optimum performance. This paper proposes a novel CAD tool for the accurate detection of pacemaker variations using machine learning models of decision tree, SVM, random forest, and AdaBoost. The models have been used to extract radiomics features in terms of textures and then screened by their Relief-F scores for selection and ranking to be classified into nine groups consisting of up to 250 radiomics features. Ten best features were fed to the machine learning models. The R-wave dataset achieved a maximum test performance accuracy of 97.73% with four features in the random forest model. The T-wave dataset achieved a maximum test performance accuracy of 96.59% with three features in the SVM model. Our experimental results demonstrate the system's robustness, which can be developed as an early and accurate detection system for pacing-induced cardiomyopathy.

## 1. Introduction

Cardiac pacemakers are used in the treatment of patients with symptomatic bradycardia. The pacemaker paces the heart at a predetermined rate to maintain uninterrupted cardiac activity [1]. Usually, pacemaker lead will be connected to right atrium (RA) and right ventricle (RV) in case of dual-chamber pacemaker implantation and to RV alone in single-chamber pacemaker implantation. This alters the route of formal conduction across the myocardial cells. The cell-to-cell conduction transmission in pacing delays the activation of selected intraventricular myocardial activation [2, 3]. This leads to electrical and mechanical desynchrony in the ventricular segmental function. These temporal alterations in myocardial function status are dependent on the pacing site at the RV cavity, which alters the physiology of ventricular electrical activation. Cardiac desynchrony can be determined by the different echocardiographic techniques including M-mode, Doppler method, tissue Doppler method, and speckle tracking echocardiography which gives subjective measures and often requires expertise in the field. Interventricular desynchrony can be determined by the Doppler method, which denotes a significant difference between RV and LV preejection period where the activation of LV is delayed considerably. RV pacing is also responsible for LV intraventricular desynchrony, which in turn increases myocardial wall stress and leads to LV failure on long-term follow-up [4–6]. Echocardiographic studies have proven the increased ventricular cavity dimensions postpacemaker implantation which were apparent after 6 months of implantation [7]. In the long term, this results in cardiac dysfunction, specifically impairing LV function and called pacemaker-induced cardiomyopathy [8, 9]. Computer-aided diagnosis (CAD) plays a crucial role in developing noninvasive techniques which can detect the subtle variations in pacemaker functions in their early stage using heart ultrasound (US) images. Creating such a CAD system requires a diverse and huge database to reach optimum performance. This study is aimed at developing an automated system for the classification of pacemaker-implanted patients from healthy control using US images of left ventricular systolic function. To the best of our knowledge, it is the first method developed in classifying the ultrasound images of the heart in pacemaker-implanted patients and healthy patients with normal left ventricular systolic function and further detecting the variations in pacemaker functions in its early stage using heart ultrasound images. The paper is organized as follows: Section 1: Introduction, Section 2: Methodology, Section 3: Experimental Results, and Section 4: Discussion.

## 2. Methodology

This study is aimed at classifying the ultrasound images of a heart in pacemaker-implanted patients and in healthy patients with normal left ventricular systolic function to see the overall changes from the end diastole to end systole between the two groups using automated detection tool, which is aimed at systematically extracting and processing the 250+ features of the ultrasound by employing the Relief-F feature selection method and processing through decision tree, AdaBoost, random forest (RF), and Support Vector Machine (SVM). The detailed architecture of the proposed model is given in Figure 1.

### 2.1. Data Acquisition

A total of 64 ultrasound images of pacemaker-implanted patients and 46 images of healthy individuals were included in the study. The study was conducted after obtaining the institutional ethical clearance, and informed consent was taken from each participant. Patients who underwent permanent pacemaker implantation prior to 6 months were included in the study. At the same time, healthy individuals attending the outpatient department for routine health checks were served as controls. Patients with left ventricular dysfunction, ischemic heart disease, and cardiomyopathy were excluded from the study. Since the pacemaker interferes with the activation of the intraventricular myocardial segment, we drew 2 frames from one cardiac cycle loop, corresponding to end diastolic and end systolic phase that are consistent with Q wave and Peak of T-wave of ECG signals from both the study groups. Sample ultrasound images of the healthy and control group are given in Figure 2.

### 2.2. Radiomics Feature Extraction

Up to 250 radiomics features from nine groups were extracted from each heart ROI: (a) histogram (9 features) [10]: mean, variance, skewness, kurtosis, percentile (perc) K% (K = 1, 10, 50, 90, and 99); (b) autoregressive model (5 features) [11]: teta1, 2, 3, 4, and sigma; (c) gradient (5 features) [10]: percentage of nonzero pixels (NonZeros) in gradients image, kurtosis, skewness, variance, and mean; and (d) histogram of oriented gradients (28 features) [12]: occurrence of gradient orientations. It is calculated for three different angular bins, 4 bins (O4b0 to Ob4b3, 4 features), 8 bins (O8b0 to O8b7, 8 features), and 16 bins (O16b0 to O16b15, 16 features); (e) Gabor (24 features) [13]: the magnitude of Gabor transform with different sizes of Gaussian envelope: 0 (H), 45 (Z), 90 (V), and 135-degree (N). Gabor features names are acronymized as follows: “Gab” followed by a size of Gaussian envelope and direction. For instance, Gab4H represents the magnitude of Gabor transform with Gaussian envelope size of 4 in the horizontal direction; (f) wavelet (24 features) [14]: energy of six subbands (S1 to S8) in three different frequency channels: low-high (LH), high-low (HL), and high-high (HH). Harr mother wavelet family was used for image decompositions. Wavelet feature names are acronymized as follows: “Haar” followed by a level of subband and channel. For instance, HaarS1HH stands for energy of decomposed image in the first subband and the HH-channel; (g) gray-level run-length matrix (GRLM, 28 features) [15]: direction: (0 (H), 45 (Z), 90 (V), and 135-degree (N)). The GRLM features are run-length nonuniformity (RLNonUni), gray-level nonuniformity (GLevNonUn), long run emphasis (LngREmph), short run emphasis (ShrtREmph), fraction, normalized run-length nonuniformity (NRLNonUni), and normalized gray-level nonuniformity (NGLevNonUni). GRLM features names are acronymized by the desired direction followed by the name of a specific GRLM feature. For instance, HGLevNonUn means gray-level nonuniformity feature in the horizontal direction. (h) Gray-level cooccurrence matrix (GLCM, 11 features) [16]: specific intensities in specific distance (1 in this study) and in all directions. The GLCM features are contrast, correlation (Correlat), sum of squares (SumOfSqs), inverse difference moment (InvDfMom), difference entropy (DifEntrp), difference variance (DifVarnc), entropy, angular second moment (AngScMom), sum entropy (SumEntrp), sum average (SumAverg), and sum variance (SumVarnc). (i) Local binary patterns (LBP, 116 features) [17]: compare intensity of pixels within a specific window size according to overcomplete (Oc), transition (Tr), and center-symmetric (Cs) algorithms. LBP features were calculated within four (4n) window size for Tr (Tr4n0 to Tr4n15, 16 features) and Oc (Oc4n0 to Oc4n15, 16 features) algorithms. For Cs algorithm, three window sizes of four (Cs4n0 to Cs4n3, 4 features), eight (Cs8n0 to Cs4n15, 16 features), and twelve (Cs12n0 to Cs4n63, 64 features) were used.

### 2.3. Feature Selection and Ranking

All radiomics features were checked for normality distribution using the Kolmogorov-Smirnov test. In addition, the independent-sample *t*-test was used to compare radiomics features among groups. The SPSS software (BM SPSS Statistics 22) was used for statistical analysis, and *P* < 0.05 was considered significant.

The Relief-F feature selection method was used for feature reductions, i.e., removing irrelevant and redundant significant features and selecting the best significant features to classify the groups (Tables 1 and 2). Relief [18] is a filtering algorithm that estimates attributes' quality based on how well their values differ between close instances. Relief-F [19] is an extension of relief, which systematically handles noisy and incomplete and multiclass data.

The performance of each model in both training and testing phases is evaluated, and sensitivity, specificity, accuracy, and area under the ROC curve are reported. This study assigns positive and negative cases to the patients and controls, respectively.

### 2.4. Classification

Classification is the process of identifying the true label of the test samples based on the best features defined by Relief-F method. This study used four classification algorithms, namely, decision tree, Support Vector Machine (SVM), random forest, and AdaBoost classifiers. Following are the details of the used classifiers.

#### 2.4.1. Decision Tree

Decision tree classifiers are constructed using both features and rules. Based on these decisions, better features and rules are grown. In a decision tree-based classifier, we begin with initial features and then use those data points as the basis for decisions that will help grow better features. We continue this process until our trees reach optimal size or we achieve a good set of rules [20, 21]. The tuning parameters of decision tree were set for both T- and R-wave ultrasound image analyses as follows: binary tree was used, min split subset: 5 and maximum tree depth: 20.

#### 2.4.2. Support Vector Machine (SVM)

*SVM* is a classification algorithm used when there are two classes, each of which has many attributes, but where some attributes have much more predictive value than others. Unlike a regular classifier, SVMs attempt to find a single hyperplane that separates the two classes and does so as well as possible. That is, an SVM chooses the parameters (the coefficients for the equation of the separating hyperplane) to maximize the margin between the two classes. The hyperplane is perpendicular to the origin and is found by solving an optimization problem [22]. The tuning parameters of SVM were set for both T- and R-wave ultrasound image analyses as follows: regression cost: 1, type of kernel: RBF, and numerical tolerance: 0.10.

#### 2.4.3. Random Forest

Random forest is a classifier that is constructed by aggregating several decision trees. The input variables are split up into subsets, one per tree, and then randomly assigned to their own individual trees. The resulting model is a collection of trees or a forest. When random forest is used on new data, the model is fit on a random selection of the original data, and the remaining data is used to estimate the accuracy of the fit. The accuracy is computed using various estimators, such as the Gini impurity for classification problems [23, 24]. The tuning parameters of random forests were set for T- and R-wave ultrasound image analyses, respectively, as follows: number of trees: 29 and 28, number of attributes considered at each split: 5 and 3, and depth of individual trees: 8 and 5.

#### 2.4.4. AdaBoost

AdaBoost is a machine learning algorithm that identifies the informative variables within a predictive model [25]. In machine learning, there are a lot of variables whose values contribute to the prediction of a target variable. Ideally, we want to use all those variables in our predictive model. But there are inherent problems with overfitting, which is the situation where the model learns the noise in the data instead of the predictive relationships. The overfitting problem is addressed by using a subset of variables called a hypothesis and adding a penalty within the loss function to ensure that the size of the hypothesis is less than or equal to a certain number. You can think of AdaBoost as a family of algorithms for selecting a good subset of the variables. The algorithm for AdaBoost is very simple in principle but results in a very complex algorithm to implement. The tuning parameters of AdaBoost were set for both T- and R-wave ultrasound image analyses as follows: base estimator: tree, number of estimators: 50, learning rate: 0.1, and regression loss function: square.

## 3. Experimental Results

The proposed model is tested on a set of 64 patients with 46 control subjects. Up to 250 radiomics features from 9 groups (histogram, AR model, gradient, etc.) were extracted from each ultrasound images. This process is implemented for obtaining both R-wave and T-wave data individually for the same dataset. The SPSS software (BM SPSS Statistics 22) was used for statistical analysis, and *P* < 0.05 was considered significant. The Relief-F feature selection method was used for cutting redundancy and selecting the best features. Based on the Relief-F scores, the ten best radiomics features of R-wave and T-wave ultrasound images were obtained (Tables 1 and 2). The ten best features were then fed to 4 machine learning classifiers (listed in Section 2.4) for final classification of the radiomics groups. All machine learning models were trained with 80% of data (50 patients and 38 controls) using the leave-one-out cross-validation strategy. The remaining 20% of data (14 patients and eight controls) was used for the testing phase.

The initial number of selected features is set to 1, and the number of selected features is increased one by one to reach the best performance of each machine learning model. As illustrated in Figure 3, the R-wave dataset achieved a maximum test performance accuracy of 97.73% with 4 features in the random forest classifier, and the T-wave dataset achieved a maximum test performance accuracy of 96.59% with 3 features in the SVM, as illustrated in Figure 4. The feature space of the best radiomics feature combinations of R-wave and T-wave ultrasound images for random forest and support vector machine classifiers is shown in Figure 5. The models were implemented for both R-wave and T-wave datasets to obtain values for specificity, area under the curve (AUC), sensitivity, and accuracy (Tables 3 and 4). SVM yielded a deviation in percentage accuracy of 1.14% between training and testing for R-wave, and random forest yielded a deviation in percentage accuracy of 0% between training and testing for T-wave (Tables 3 and 4).

## 4. Discussion

The study's main goal is to develop a computer-aided diagnostic tool for assessing pacemaker effects and its long-term changes in contrast to healthy individuals using ultrasound images. In the current study, ultrasound images of 64 patients and 46 control subjects were used to identify the variations between healthy and pacemaker-implanted patients. The automated detection tool was used to systematically extract and process 250+ features of the ultrasound by employing the Relief-F feature selection method. The corresponding ten best features with Gabor and gradient ranking among the top two features (Tables 1 and 2) extracted were fed into four classification models (random forest, SVM, AdaBoost, and decision tree) with varying results. All machine learning models were trained with 80% of the data, and 20% was used for testing. Within the R-wave datasets, the random forest classifier achieved the maximum performance accuracy of 97.73% with four features, followed by 96.59% with the SVM model, and in the T-wave dataset, the SVM model achieved a maximum accuracy of 96.59% followed by 95.45% with the AdaBoost model with three features. Random forest and SVM have proven to be the more suitable models in this study which will immensely facilitate future work (Tables 3 and 4). Between the two performing models, the accuracy from training and testing was 0% with the random forest model, whereas the SVM model had a deviation of 1.14%.

The study obtained a maximum accuracy of 97.73% and a deviation in the accuracy of 0-1.14%, allowing for a robust approach to early detection to facilitate appropriate medical intervention. However, the current study draws its limitations with the use of a smaller dataset as only 20% of the best features were used for testing. Having a large dataset will not only aid in better training but also polish the model to run more efficiently, which leaves room for future development where a much larger dataset for training and testing can be implemented to improve the metrics of this model. Future works will involve developing the model further with the use of deep learning algorithms with larger datasets for higher detection accuracy.

### 4.1. Limitations

It is difficult to generalize the system because it uses the smaller dataset. Hence, we plan to extend our work by collecting more images in the future.

## 5. Conclusion

Although multiple factors can contribute to patients being at an increased risk for pacing-induced cardiomyopathy, many individuals have tolerated high-burden RV pacing for years without showing signs or symptoms. The ability to accurately identify those at the highest risk remains insufficient to this day. The proposed CAD tool demonstrates accurate and consistent results up to 97.73% for early risk indicators to assist in early detection and intervention, resulting in an appropriate treatment plan based on the severity. In the future, we would like to develop an automated system for detecting PICM using deep learning techniques by involving more subjects. In addition, we would like to create a huge database from various hospitals and develop an IoT hybrid model to achieve promising results.

## Figures and Tables

**Figure 1:** Architecture of the proposed study.

**Figure 2:** Sample images from the pacemaker case ((a) T-wave and (c) R-wave) and control set ((b) T-wave and (d) R-wave).

**Figure 3:** Plot of accuracy versus different best significant radiomics feature combinations of R-wave ultrasound images using Relief-F method for (a) decision tree, (b) Support Vector Machine, (c) random forest, and (d) AdaBoost classifiers.

**Figure 4:** Plot of accuracy versus different best significant radiomics feature combinations of T-wave ultrasound images using Relief-F method for (a) decision tree, (b) Support Vector Machine, (c) random forest, and (d) AdaBoost classifiers.

**Figure 5:** Feature space of the best radiomics feature combinations of R-wave ultrasound images and T-wave ultrasound images. (a) Random forest and (b) Support Vector Machine classifiers.

**Table 1:** The best 10 radiomics features of R-wave ultrasound images obtained by Relief-F method with their scores.

Group	Rank	Features	Relief-F score
Gabor	1	Gab8V	0.273
	2	Gab8H	0.196
Gradient	3	Variance	0.127
Gabor	4	Gab6V	0.124
Local binary patterns	5	Oc4n10	0.095
	6	Oc4n4	0.094
	7	Cs12n47	0.092
Gabor	8	Gab6Z	0.091
	9	Gab6N	0.087
Cooccurrence matrix	10	DifVarnc	0.084

**Table 2:** The best 10 radiomics features of T-wave ultrasound images obtained by Relief-F method with their scores.

Group	Rank	Features	Relief-F score
Gabor	1	Gab8V	0.252
	2	Gab8H	0.165
	3	Gab6N	0.130
	4	Gab6V	0.129
	5	Gab6Z	0.117
Gradient	6	Variance	0.104
Wavelet	7	HaarS2HL	0.083
Gabor	8	Gab4H	0.081
Histogram of oriented gradients	9	O16b8	0.080
Local binary patterns	10	Cs8n9	0.079

**Table 3:** Performance of four classifiers under the best radiomics feature combination of R-wave ultrasound images in the training and test datasets.

Model	Sensitivity (%)	Specificity (%)	Accuracy (%)	AUC
Decision tree				
Training	92.00	94.74	93.18	0.912
Test	92.86	87.50	90.91	0.902
SVM				
Training	100	92.11	96.59	0.992
Test	100	87.50	95.45	0.929
Random forest				
Training	100	94.74	97.73	0.988
Test	100	87.50	95.45	0.964
AdaBoost				
Training	94.00	97.37	95.45	0.901
Test	92.86	87.50	90.91	0.909

**Table 4:** Performance of four classifiers under the best radiomics feature combination of T-wave ultrasound images in the training and test datasets.

Model	Sensitivity (%)	Specificity (%)	Accuracy (%)	AUC
Decision tree				
Training	92.00	86.84	89.77	0.883
Test	100	87.50	95.45	0.924
SVM				
Training	100	92.11	96.59	0.999
Test	100	87.50	95.45	0.955
Random forest				
Training	100	89.47	95.45	0.955
Test	100	87.50	95.45	0.945
AdaBoost				
Training	100	89.47	95.45	0.947
Test	92.86	87.50	90.91	0.909

## Data Availability

No data were used to support this study.

## Additional Points

*Highlights of the Research Work.* (i) The system uses the leave-one-out cross-validation strategy. (ii) It uses only four features to achieve maximum classification accuracy. (iii) To the best of our knowledge, this is the first work to detect the variations in pacemaker functions in its early stage.
